RETRACTED

# Exogenous supplement of N-acetylneuraminic acid improves macrophage reverse cholesterol transport in apolipoprotein E-deficient mice

**DOI:** 10.1186/s12944-019-0971-1

**Published:** 2019-01-24

**Authors:** Pengbo Hou, Shumei Hu, Jin Wang, Zixun Yang, Jiayu Yin, Guanghai Zhou, Shoudong Guo

**Affiliations:** 1 Research Center on Life Sciences and Environmental Sciences, Harbin University of Commerce, Harbin, 150076 China; 2 Institute of Lipid Metabolism and Atherosclerosis, Innovative Drug Research Centre, School of Pharmacy, Weifang Medical University, 7166# Baotongxi Street, Weifang, 261053 Shandong Province China; 3 Taishan Medical University, Taian, 271000 China

**Keywords:** Istope tracing; sialic acid, Atherosclerosis, High-fat diet

## Abstract

**Background:**

N-acetylneuraminic acid (NANA) is the major form of sialic acid in mammals, and the plasma NANA level is increased in patients with cardiovascular diseases. Exogenous supplement of NANA has been demonstrated to reduce hyperlipidaemia and the formation of atherosclerotic lesions; however, the underlying mechanisms have not yet been clarified. The aim of this study is to investigate whether exogenous supplement of NANA improves reverse cholesterol transprot (RCT) in vivo.

**Methods:**

Apolipoprotein E-deficient mice fed a high-fat diet were used to investigate the effect of NANA on RCT by [^3^H]-cholesterol-loaded macrophages, and the underlying mechanism was further investigated by various molecular techniques using fenofibrate as a positive control.

**Results:**

Our novel results demonstrated that exogenous supplement of NANA significantly improved [^3^H]-cholesterol transfer from [^3^H]-cholesterol-loaded macrophages to the plasma (an increase of > 42.9%), liver (an increase of 35.8%), and finally to the feces (an increase of 50.4% from 0 to 24 h) for excretion in apolipoprotein E-deficient mice fed a high-fat diet. In addition, NANA up regulated the protein expression of ATP-binding cassette (ABC) G1 and peroxisome proliferator-activated receptor α (PPARα), but not the protein expression of ABCA1and scavenger receptor B type 1 in the liver. Therefore, the underlying mechanism of NANA in improving RCT may be partially due to the elevated protein levels of PPARα and ABCG1.

**Conclusion:**

Exogenous supplement of NANA improves RCT in apolipoprotein E-deficient mice fed a high-fat diet mainly by improving the protein expression of PPARα and ABCG1. These results are helpful in explaining the lipid-lowering effect of NANA.

## Background

Sialic acids are found at terminal positions of glycoconjugate, and play important roles in various biological and pathological processes [1, 2]. N-acetylneuraminic acid (NANA) is the major type of sialic acid in mammals [3]. The total sialic acid level is increased in the plasma of patients with cardiovascular disease (CVD), and it has been reported as a biomarker of the sustained inflammatory response [1, 2]. Interestingly, recent studies have indicated that sialic acids have antioxidant activities [4–6], and exogenous NANA could be employed as a therapeutic option in some diseases [7].

RETRACTED

Hyperlipidaemia is one of the major risk factors for the development and progression of CVD, and reverse cholesterol transport (RCT) is believed to facilitate it [8]. Glomset et al. originally proposed the concept of RCT in 1973 [9]. RCT is a physiological process in which excess peripheral cholesterol is transported by high-density lipoprotein (HDL) or non-HDL to the liver for excretion into the bile and feces. Tang et al. proposed a new model, the named cholesterol transport system, which involves cholesterol absorption in the small intestine, cholesterol influx and esterification in peripheral cells and transintestinal cholesterol excretion [10]. A previous study reported that exogenous NANA can partially ameliorate atherosclerosis in apolipoprotein E-deficient (*apoE*^*−/−*^) mice partially by lowering the level of lipids [11]. Furthermore, synthesized quercetin7-O-sialic acid benefits cholesterol efflux in vitro [12]. We speculate that the increased sialic acids may underlie the compensatory mechanism through its lipid-lowering role in regulating RCT in patients with CVD.

The aim of this study is to investigate whether exogenous supplement of NANA improves RCT in *apoE*^*−/−*^ mice fed a high-fat diet and to elucidate the underlying mechanism.

## Methods

### Materials

RAW 264.7 macrophages were purchased from Shanghai BoYao Biological Technology Co., Ltd. (Shanghai, China). N-acetylneuraminic acid (NANA, 98.5% purity) was a product of Wuxi AccoBio Biotechnology Incorporated (Wuxi, China). Dulbecco’s modified Eagle’s medium (DMEM) and foetal bovine serum (FBS) were from Gibco (BRL, Gaithersburg, MD, USA). Complete protease inhibitor cocktail tablets were purchased from Roche (Schweiz, Germany). RIPA lysis buffer was a product of Solarbio (Beijing, China). Rabbit polyclonal antibody against ATP binding cassette (ABC) G1, mouse monoclonal antibody against ABCA1 and rabbit monoclonal antibody against scavenger receptor B type 1 (SR-B1) were from Abcam (Cambridge, MA, USA). Peroxisome proliferator-activated receptor α (PPARα) and cholesterol 7 alpha-hydroxylase A1 (CYP7A1) were purchased from Santa Cruz Biotechnology (Santa Cruz, CA, USA). Enhanced chemiluminescence (ECL) kits were purchased from Thermo Scientific Pierce (Rockford, IL, USA). All reagents used in this study were of analytical grade.

RETRACTED

### Animals

Fifteen *apoE*^*−/−*^ mice with a C57BL/6 genetic background (male, 20 ± 2 g body weight) were purchased from Beijing HFK Bioscience Co., Ltd. (license number: SCXK2014–0010). All-experiments were approved by the Laboratory Animal Ethical Committee of Taishan Medical University and followed the NIH Guidelines for the Care and Use of Animals. Mice were fed a high-fat diet (15% fat and 1.0% cholesterol). After acclimatization for 1 week, the mice were randomly divided into three groups, namely, the blank control group (*n* = 5, 0.9% sodium chloride by gavage, vehicle), the fenofibrate group (n = 5, 50 mg/kg/d by gavage) [13], and the NANA group (n = 5, 200 mg/kg/d NANA in the drinking water). The dose of NANA was determined as previously described [11].

### Preparation of lipoproteins

Lipoproteins were prepared using sequential ultracentrifugation as previously described [14, 15]. In brief, the plasma density was adjusted to 1.006 g/mL for ultracentrifugation at 10 °C (393,000×g for 24 h). The upper layer containing very low-density lipoproteins was removed, and the density was re-adjusted to 1.063 g/mL for ultracentrifugation at 393,000×g for an additional 24 h to obtain the upper layer containing low-density lipoproteins (LDL) in the upper layer. The density was re-adjusted again to 1.21 g/mL for ultracentrifugation at 393,000×g for an additional 48 h to obtain the upper layer containing high-density lipoproteins (HDL). EDTA-2Na (0.1%, *w*/*v*) was added to chelate the metal ions, thereby reducing oxidation during ultracentrifugation. The protein content of the fractions was determined by the Bradford method. The LDL and HDL fractions were stored at 4 °C until use.

### Preparation of [^3^H]-cholesterol-loaded macrophages

[^3^H]-cholesterol (5 μCi/mL) and oxidized LDL (100 μg/mL) were mixed and pre-incubated at 37 °C for 30 min. RAW 264.7 macrophages were cultured in DMEM supplemented with 10% FBS. The cells were harvested after incubation for 48 h and intraperitoneally injected into mice (5.5 × 10^5^ cells containing 6.0 × 10^4^ cpm in 0.5 mL of DMEM per mouse) [12, 15].

### In vivo reverse cholesterol transport assay

After treatment with NANA or fenofibrate for 6 weeks, mice were injected with [^3^H]-cholesterol-loaded macrophages. Thereafter, blood (100 μL) was sampled from the retro-orbital sinus at 0, 12, 24 and 48 h, and faeces were collected every 24 h. The animals were euthanized, and the livers were collected.

Liver (0.3 g) or faeces were homogenized in a hexane/isopropanol (3:2, *v*/v) solution, and the mixtures were placed on a shaker for 12 h at room temperature. Thereafter, the mixture was centrifuged at 5000×g for 15 min, and the supernatant was kept for measurement. Prepared samples were transferred into 5.0 mL scintillation vials, and 4.0 mL of HIONIC FLUOR™ complete LSC-cocktail (PerKinElmer, Inc., Waltham, MA, USA) was then added and mixed well. The scintillation vials were counted on a SN-6930B type liquid scintillation counter (BECKMAN, USA). The results were expressed as a percentage of injected [^3^H]-cholesterol or directly by counts per minute (CPM) [15].

RETRACTED

### The cholesterol efflux assay in vitro

This experiment was performed as suggested by Low et al with some modifications [16]. In brief, Raw 264.7 macrophages were plated into 24-well plates at a final density of 1 × 10^5^ cells per well. Six hours later, the culture medium was discarded and cells were gently washed with PBS 3 times. Then, 600 μL of DMEM containing 1% FBS and 1 μCi/mL [^3^H]-cholesterol was added to each well and incubated for an additional 24 h. After the incubation, the medium containing [^3^H]-cholesterol was removed, and the cells were gently washed with PBS 3 times. Cells were treated with 500 μL of DMEM containing 1% FBS in the presence or absence of FF (5.0 μM) or NANA (5.0 μM) for 4 h, and 100 μL of HDL (final concentration of 20 μg/mL) was then added and incubated for an additional 6 h. The culture medium was collected in 1.5-mL microfuge tubes and centrifuged at 14,000 rpm for 10 min at room temperature to remove cellular debris. Cells in the well were treated with 1 mL of hexane/isopropanol (3:2, *v*/v) for 30 min at room temperature. The extract was transferred into 1.5-mL microfuge tubes and centrifuged as described above. Next, 200 μL of medium or cell extract was used for measuring [^3^H]-cholesterol, as described above. The percentage of [^3^H]-cholesterol was calculated as follows: efflux% = [CPM of the media/(CPM of the media + CPM of the cell extract)] × 100%.

### Protein isolation, electrophoresis, and western blotting

Total proteins from the liver or aorta were extracted using RIPA lysis buffer with complete protease inhibitor according to the manufacturer’s instructions. Equal amounts of protein were subjected to 12% or 10% SDS-PAGE and transferred onto Polyvinylidene fluoride membranes by electroblotting. After blocking in Tris-buffered saline containing 0.1% Tween-20 and 5% nonfat dry milk for 2 h at room temperature, the membranes were incubated with primary antibodies overnight at 4 °C. After washing 3 times, the membranes were incubated with horseradish peroxidase-conjugated secondary antibodies for 2 h at room temperature. Immunoblots were revealed by enhanced chemiluminescence reaction and visualized using a high performance chemiluminescence film. Densitometry analysis was conducted using Image-Pro Plus software version 6.0 (Media Cybernetics Corp, Bethesda, MD, USA) and normalized by housekeeping protein β-actin [12, 14].

RETRACTED

### Data analysis

All of the bioassay results were expressed as the mean ± standard deviation (*SD*) for at least three independent experiments. Statistical analysis was performed using one-way analysis of variance (ANOVA) followed by Tukey’s test. Differences were considered to be significant at a *P* < 0.05.

## Results

### NANA lowers the total cholesterol level and improves reverse cholesterol transprot in *apoE*^*−/−*^ mice

Compared to the control group, NANA significantly lowered the plasma TC level in the *apoE*^*−/−*^ mice fed a high-fat diet (Fig. 1a, approximately 19.0%, *P* < 0.05). Equally important, NANA increased the transfer rate of [^3^H]-cholesterol from the injected macrophages to the plasma, and this was most significant at the 12 h time point (increased approximately 1.3-fold compared to the control, Fig. 1b). Furthermore, [^3^H]-cholesterol transported to the liver for excretion increased approximately 35.8% in mice treated with NANA compared to those treated with vehicle (*P* < 0.05, Fig. 1c). As a consequence, [^3^H]-cholesterol excreted in the faeces of treated mice was significantly elevated (~ 50.4%) from 0 to 24 h compared with untreated mice (Fig. 1d). Additionally, fenofibrate significantly affected [^3^H]-cholesterol transport from the injected macrophages to the plasma from 0 to 24 h and 24 to 48 h, (*P* < 0.05, Fig. 1b), liver (~ 35.5%, *P* < 0.05, Fig. 1c) and feces (~ 64.0% from 0 to 24 h and ~ 42.4% from 24 to 48 h, Fig. 1d). However, there was no difference in the improvement of RCT between mice of NANA and fenofibrate groups.

**Fig. 1:** NANA lowers the TC level and improves reverse cholesterol transport in *apoE*^*−/−*^ mice (*n* = 5). **a**, NANA lowers the plasma TC level in the *apoE*^*−/−*^ mice; **b**, NANA increases the transfer rate of [^3^H]-cholesterol from the injected fat-laden macrophages to the plasma of *apoE*^*−/−*^ mice; **c**, [^3^H]-cholesterol in the liver of *apoE*^*−/−*^ mice 48 h after injection; **d**, [^3^H]-cholesterol in the faeces of *apoE*^*−/−*^ mice. BC: blank control; FF: fenofibrate; NANA: N-acetylneuraminic acid. Data are expressed as the means ± SD. * *p*<0.05 vs BC group; ** *p*<0.01 vs BC group

In this study, NANA significantly improved the protein expression of PPARα (approximately 32.3%) and ABCG1 (approximately 34.1%) in the liver (*P* < 0.05, Fig. 2a and b); however, it did not affect the protein expression of SR-BI and CYP7A1 in the liver of *apoE*^*−/−*^ mice (Fig. 2c and d). In addition, fenofibrate significantly improved the protein expression of PPARα (~ 82.7%) and ABCG1 (~ 41.9%) in the liver (*P* < 0.05, Fig. 2a and b), but not the protein expression SR-BI and CYP7A1 in the same organ (Fig. 2c and d).

RETRACTED

**Fig. 2:** NANA improves the protein expression of PPARα and ABCG1 in the livers of *apoE*^*−/−*^ mice (*n* = 3). **a**, protein expression of PPARα and densitometric quantification; **b**, protein expression of ABCG1 and densitometric quantification; **c**, protein expression of SR-BI and densitometric quantification; **d**, protein expression of CYP7A1 and densitometric quantification. BC: blank control; FF: fenofibrate; NANA: N-acetylneuraminic acid. Data are expressed as the means ± SD. * *p*<0.05 vs BC group; ** *p*<0.01 vs BC group

### NANA improves cholesterol efflux and ABCG1 expression in vitro

Both NANA and fenofibrate at concentrations of 5.0 μM improved [^3^H]-cholesterol efflux; however, the effect of NANA was weaker than that of fenofibrate (*P* < 0.01, Fig. 3a). To investigate the underlying mechanism, the protein levels of ABCA1, ABCG1 and SR-BI were measured. As shown in Fig. 3 B-D, NANA significantly increased the protein expression of ABCG1 (~ 31.6%, *P* < 0.05), but not that of ABCA1 and SR-BI in the treated macrophages compared to untreated cells. Furthermore, fenofibrate increased the protein expression of ABCG1 in treated macrophages (~ 61.7%, *P* < 0.01).

**Fig. 3:** NANA improves cholesterol efflux and increases the protein expression of ABCG1 in RAW264.7 macrophages (*n* = 3). **a**, NANA improves [^3^H]-cholesterol efflux; **b**, protein expression of ABCA1 and densitometric quantification; **c**, protein expression of ABCG1 and densitometric quantification; **d**, protein expression of SR-BI and densitometric quantification. BC: blank control; FF: fenofibrate; NANA: N-acetylneuraminic acid. Data are expressed as the means ± SD. * *p*<0.05 vs BC group; ** *p*<0.01 vs BC group; ^##^ *p*<0.01 vs FF group

## Discussion

RCT hauls excess cholesterol from peripheral cells, especially macrophages, to the liver for excretion. This study revealed for the first time that NANA significantly improved RCT in vivo using [^3^H]-cholesterol, with the elevated protein levels of PPARα and ABCG1 possibly contributing to the underlying mechanism.

In a previous study, we demonstrated that NANA reduced hyperlipidaemia and lipid accumulation in the liver and aorta in *apoE*^*−/−*^ mice fed a high-fat diet [11]. It is interesting to investigate whether the lipid-lowering effect of NANA is related to RCT. The results of this study showed that NANA significantly improved RCT in vivo, which has never been shown before (Fig. 1). It is acknowledged that apoA1 and HDL are major acceptors of peripheral cholesterol [17, 18]. Previously, NANA was reported to improve the content of apoA1 in the plasma and ABCA1 in the liver [11], which was beneficial to the first step of RCT. This study further indicated that NANA might benefit RCT by improving the transport of cholesterol from peripheral cells to HDL. It is also known that SR-BI mediates cholesterol efflux from macrophages to extracellular HDL. However, our results indicated that NANA showed no effect on the protein expression of SR-BI [17, 18]. Cholesterol can be delivered to the liver directly by SR-B1 and indirectly by the LDL receptor after free cholesterol has been transformed into cholesterol esters by lecithin cholesterol acyltransferase. However, our results indicated that NANA showed no significant influence on the protein expression of SR-BI and LDLR in the liver. Therefore, NANA improves RCT by activating cholesterol efflux from peripheral cells to the plasma. Furthermore, ABCG5 is an important mediator involved in the secretion of cholesterol from the liver and small intestine. In a previouse study, NANA treatment up-regulated the expression of ABCG5 in the liver and small intestine [11], which may have contributed to the increase of [^3^H]-cholesterol in the faeces of *apoE*^*−/−*^ mice. In addition, CYP7A1 has an important role in cholesterol metabolism; it converts cholesterol to 7-alpha-hydroxycholesterol, the first and rate-limiting step in bile acid synthesis. Our results indicated that NANA showed no significant effect on the protein expression of CYP7A1, suggesting that NANA may have no impact on the transformation of cholesterol to bile acid.

RETRACTED

In this study, macrophages were used to investigate whether NANA could directly influence the expression of proteins involved in the first step of RCT. As expected, NANA significantly affected the protein expression of ABCG1. However, this in vitro study may not reflect the in vivo situation, because NANA is likely to improve cholesterol metabolism by influencing multiple steps and factors involved in RCT, such as by acting on non-macrophage cells. In the present study, we demonstrated that NANA could up-regulate the expression of PPARa and ABCG1 to some extent. Therefore, we speculate that NANA may exert its effect on RCT by a mechanism similar to that of fenofibrate [13, 19]. However, these results must be validated by other molecular methods such as gene knockdown or knockout and chemical inhibitors. Furthermore, mouse plasma is characterized as HDL-C dominant, whereas human plasma is not HDL-C dominant. Therefore, the major limitation of the present study is that the results may not accurately reflect what is occurring in humans. We are planning is to investigate the effect of NANA in mammals, such as the guinea pig and the rabbit, whose lipid profiles are closer to that of the humans. Additionally, RCT only reflects a part of cholesterol transport and metabolism [10], and a systemic model is needed to understand the effects of NANA on cholesterol metabolism.

## Conclusion

NANA improves RCT by up regulating the protein of PPARα and ABCG1, suggesting the increased sialic acids may underlie the compensatory mechanism in patients with CVD. Further studies are needed to confirm these results in other models.

## Abbreviations

ABC: ATP-binding cassettes
apoE: Apolipoprotein E-deficient
CPM: Count per minute
CVD: Cardiovascular disease
CYP7A1: Cholesterol 7 alpha-hydroxylase A1
DMEM: Dulbecco’s modified Eagle’s medium
FBS: Feotal bovine serum
HDL: High density lipoprotein
LDL: Low density lipoprotein
NANA: N-acetylneuraminic acid
PPARα: Proliferator-activated receptor α
RCT: Reverse cholesterol transport
SR-BI: Scavenger receptor B type 1
